The article "The Effects of Occupation-Based Community Rehabilitation for Improving Activities of Daily Living and Health-Related Quality of Life of People with Disabilities after Stroke Living at Home: A Single Subject Design" was published in 2022. Journal: Occup Ther Int.

# The Effects of Occupation-Based Community Rehabilitation for Improving Activities of Daily Living and Health-Related Quality of Life of People with Disabilities after Stroke Living at Home: A Single Subject Design

**DOI:** 10.1155/2022/6657620

**Published:** 2022-03-29

**Authors:** KwangTae Moon, WanHo Jang, Hae Yean Park, MinYe Jung, JongBae Kim

**Affiliations:** ^1^Department of Occupational Therapy, College of Software Digital Healthcare Convergence, Yonsei University, Wonju, Republic of Korea; ^2^Department of Occupational Therapy, Jeonju University, Jeonju, Republic of Korea

## Abstract

**Objective:**

The aim of this study is to investigate the effect of occupation-based community rehabilitation on activity daily of living and health-related quality of life of people with disabilities after stroke at home.

**Method:**

In this study of three people with disabilities after stroke living at home, A-B-A single-subject design was used. The occupation-based community rehabilitation was implemented during the intervention phase. It included task oriented and feedback, related information education, home environment modification, and community resource network. After applying the intervention, changes in activities of daily living and health-related quality of life were evaluated by the Modified Barthel Index (MBI), the EuroQol-5 dimension (EQ-5D), and the Assessment of Motor and Process Skills (AMPS).

**Result:**

After applying the occupation-based community rehabilitation program, all three participants' daily life activities and quality of life improved. In addition, the occupational performance skills in all participants were maintained.

**Conclusion:**

It was confirmed that individual occupational-based community rehabilitation had a positive effect on the activities of daily living and quality of life improvement of the people with disabilities after stroke at home.

## 1. Introduction

Stroke is a disease that causes temporary or permanent loss of function due to blockage or rupture of blood vessels in the brain, and physical, cognitive, and mental aspects of aftereffects cause restrictions on independent daily life [1]. About 75% of stroke patients show disabilities in independent daily life abilities [2]. If dependence on daily life continues, there is a possibility that interpersonal relationships and the quality of life may deteriorate due to helplessness and depression [3].

Hospitalization for a considerable period after stroke is the most common approach for postoperative rehabilitation or intensive care for acute patients, and institution-based rehabilitation (IBR) provides expert-centered services for rehabilitation. However, this approach has limitations due to systematic discharge preparation, insufficient community integration procedures, lack of information on community services, and poor access to community services [4–6].

The article "The Effects of Occupation-Based Community Rehabilitation for Improving Activities of Daily Living and Health-Related Quality of Life of People with Disabilities after Stroke Living at Home: A Single Subject Design" was published in 2022. Journal: Occup Ther Int.

In Korea, it was recommended that community-based rehabilitation (CBR) health centers organize community early adaptation programs, rehabilitation programs for the disabled, assistance device support, and health examination support programs for the disabled. CBR managers should classify the people with disabilities into different groups based on their ability for activities of daily living and quality of life, integrate and provide community public and private resources for the health care of the people with disabilities, and continuously monitor health state to meet the needs of the disabled [7].

When providing rehabilitation in the community, occupational therapists have played a key role in evaluating and mediating daily life activities, evaluating and modifying residential environments, educating assistive device, and connecting community resources with stroke patients [8–11].

In the case of activities of daily living, a previous study showed that one of the most effective ways is to directly observe occupational performance and educate task directly [12]. In order to reduce barriers in home environment, the home environmental modification was effective in aiming to change the location of the home structure and improve the ability of the subject [13]. It has been reported that it is effective to provide integrated and personalized interventions and provide information on available community resources according to the needs and functions of the education of the stroke patient's guardian [14]. However, despite the growing need for occupational therapy other than hospitals, the participation of occupational therapists is limited due to the lack of legal grounds, poor working conditions, and payment systems. Therefore, it is timely to generate evidence by conducting a single target study that takes into account the individual characteristics of the stroke patients and the community environment.

In previous studies, it was difficult to understand in detail each report on the results of daily life performance intervention through task-oriented methods, home environmental modification, guardian education on related diseases and interventions, and information on available community resources. In the clinical setting in the real world, interventions are applied integrally rather than individually, so it is important to investigate the roles and responsibilities of the occupational therapists by integrating and applying each intervention into occupation-based community interventions. The process of designing and analyzing occupation-based community intervention as a single subject design for people with disabilities after stroke can be an important process to suggest the direction of development of the study.

The article "The Effects of Occupation-Based Community Rehabilitation for Improving Activities of Daily Living and Health-Related Quality of Life of People with Disabilities after Stroke Living at Home: A Single Subject Design" was published in 2022. Journal: Occup Ther Int.

According to these needs, occupation-based community rehabilitation is necessary to improve the daily life and quality of life of people with disabilities after stroke. The purpose of this paper is to investigate whether occupation-based community rehabilitation is effective in improving the daily life ability and quality of life of people with disabilities after stroke using a single subject design research.

## 2. Methods

This study investigated the effect of occupation-based community rehabilitation on the activities of daily living and health-related quality of life of people with stroke living at home.

### 2.1. Research Design

The A-B-A design was used as a single-subject research design. In this paper, we recruit participants for baseline phase A, intervention phase B, baseline phase A', and follow-up phase. The period of the study was 17 weeks from April to August 2020. This paper was reviewed and approved by the Yonsei University Wonju Campus Biomedical Review Committee (YUWIRB). It was performed prior to conducting the study (approval number: 1041849-202001-SB-001-02).

### 2.2. Participants

The study participants were collected and analyzed from three people with severe disabilities (grades 1 to 3 for disability) living at home after stroke. Participants in this study were recruited according to the selection and exclusion criteria among people with stroke registered in the CBR project at the public health center for four weeks. The selection criteria included (1) with a score of ≤49 in the Modified Barthel Index (MBI) or with a score of <0.660 [7]; (2) those who have passed more than 6 months from the date of stroke; (3) a person diagnosed with a stroke by a specialist; and (4) those who understood and agreed to the purpose of the study were included. The exclusion criteria included (1) people with no guardians or other overlapping disabilities; (2) people who participated in other rehabilitation studies or drug experiments; and (3) people who could not communicate were excluded.

## 3. Measures

### 3.1. Modified Barthel Index (MBI)

The MBI was used as a tool to evaluate functional changes in stroke patients and to evaluate daily life behavior independence, and in 1989, Shah et al. [15] modified and supplemented the Barthel Index to evaluate daily life activities of chronically ill patients, and its validity and reliability have been proven [16]. MBI consists of a total of 10 items, 7 items for self-care index and 3 items for mobility index. Evaluation is conducted through guardian investigation or observation. The total score range is from 0 to 100, with a total score from 0 to 24, severity from 25 to 49, a middle from 50 to 74, a middle from 75 to 90, and a minimum from 91 to 99.

The article "The Effects of Occupation-Based Community Rehabilitation for Improving Activities of Daily Living and Health-Related Quality of Life of People with Disabilities after Stroke Living at Home: A Single Subject Design" was published in 2022. Journal: Occup Ther Int.

### 3.2. EuroQol-5 Dimension (EQ-5D)

The EQ-5D, developed by EuroQol Group, is a measurement tool for overall health and is evaluated in the form of a subject survey. EQ-5D is an indicator of health-related quality of life, which can be used to evaluate nondisabled and health-related quality of life as well as disabled people and is expected to identify vulnerable groups along with health policy evaluation [17]. It consists of a total of five areas: mobility, self-management, daily activities, pain/comfort, and anxiety/depression. Health-related quality of life scores are calculated from 1 to -1 by applying weights to each value measured for each domain. Complete health status is 1 point, and health status worse than death is -1. Health-related quality of life scores were calculated by applying weight calculation equations according to Lee et al. [18].

### 3.3. Assessment of Motor and Process Skills (AMPS)

AMPS is a standardized tool centered on subjects to evaluate motor skills and process skills, which are observed during daily life activities, rather than just evaluating the cognitive or physical damage of stroke clients [19]. It consists of a total of 7 items, divided into positioning, maintaining objects in hands, moving oneself and objects, continuing performance, applying knowledge, organizing space and objects, and controlling performance. Each AMPS technology item is scored on a four-step classification basis, and each step is classified as 4 = competent, 3 = questionable, 2 = ineffective, and 1 = severely limited occupational performance technology. As a result of the query of occupational performance, the raw score of each technical item is entered into the Occupational Therapy Assessment Package (OTAP) software provided by CIOTS, and the OTAP software considers the evaluator's roughness, task difficulty, and item difficulty. The ability ranges from -3.0 to 4.0, and the ability to live without help in the community is based on 2.0 in athletic skills and 1.0 or more in processing skills. The clinically significant change in competency is 0.3 to 0.4, and the statistically significant change is 0.5 or more, which is interpreted as an improvement in occupational performance. AMPS inspection-reinspection reliability is 0.81 and 0.71 when only one task is performed, and the areas of exercise technology and processing technology are 0.91, and 0.85, respectively, showing higher reliability in two or more tasks [20].

The article "The Effects of Occupation-Based Community Rehabilitation for Improving Activities of Daily Living and Health-Related Quality of Life of People with Disabilities after Stroke Living at Home: A Single Subject Design" was published in 2022. Journal: Occup Ther Int.

## 4. Procedures

### 4.1. Baseline Phase A

During 5 sessions in three weeks in baseline phase A, the researcher dropped in on each participant's home. The researcher observed the difficult and good activities chosen by the participants for 15 to 20 minutes and observed and recorded changes in the frequency of occupational performance by session. The participants signed and complied with the occupation contract before starting the task, and the task was completed after 5 minutes per occupation. MBI, EQ-5D, and AMPS were evaluated before baseline phase A.

### 4.2. Baseline Phase B

During 14 sessions in seven weeks in intervention phase B after the end of baseline phase A, researcher visited each participant's home for the experiment. In the first session, preevaluation results were explained, and individual customized methods were trained for participants and caregivers. The contents of the education consisted of analyzing the daily life observed in advance, revising and proposing in a beneficial direction to improve effective daily life and occupational performance ability, and presenting tasks to improve daily life ability. The task was performed daily like a routine habit, and the participants recorded the task in the task notebook and delivered it to the researcher to receive feedback every session. MBI, EQ-5D, and AMPS were evaluated after baseline phase B.

### 4.3. Baseline Phase A'

During 5 sessions in three weeks in baseline phase A', in the same way as in the baseline phase A, the researcher called on the participant's home to observe the participant's daily life performance, and in the final term, the participant's future was consulted.

### 4.4. Follow-up Phase

In order to find out whether occupational-based community rehabilitation affects the daily life and quality of life of the disabled, a follow-up phage was conducted four weeks after the baseline A'. MBI, EQ-5D, and AMPS were evaluated in follow-up phase.

## 5. Independent Variable (Occupational-Based Community Rehabilitation Program)

This study used the occupation-based community rehabilitation program to improve the daily life and quality of life of people with stroke. Occupation-based community rehabilitation program consisted of task-oriented methods and feedback, home environmental modification, related information and education, and linking local resource.

### 5.1. Task-Oriented Methods and Feedback

In this study, the task-oriented approach is a training method focusing on special functional tasks that combine musculoskeletal or nervous systems and provides the participant's occupation-based daily life as a task rather than repeatedly practicing normal patterns. In order to build tasks based on the occupation of each participant, the researcher prioritized meaningful activities for each topic according to OTIPM. However, if the participant performed the task for the first time or failed to perform it independently, it was possible to learn how to perform the task accurately by referring to the error-free fourth stage of learning by Thivierge et al. [21]. The task difficulty and the amount of help changed according to the participant's degree of occupational performance.

The article "The Effects of Occupation-Based Community Rehabilitation for Improving Activities of Daily Living and Health-Related Quality of Life of People with Disabilities after Stroke Living at Home: A Single Subject Design" was published in 2022. Journal: Occup Ther Int.

### 5.2. Home Environmental Modification

Home environmental modification was performed to improve participants' activities of daily living. After checking the participants' spatial environment, the researcher changed the location of the structure and installed tools to prevent safety accidents to lower environmental barriers and increase convenience [22]. If necessary, it was proceeded through a contract with the lessor. The researcher applied and modified it to suit the participants to improve the performance of daily life in the changed family environment during the study period.

### 5.3. Related Information Education

Local community information and medical welfare resources tailored to the characteristics and needs of the participants were provided, and if necessary, they were directly linked to local resources. The linkage of local resources was able to meet the complex needs of medical welfare targets by identifying the complex needs of the participant s and finding and linking community services accordingly. The researcher checked the socioeconomic aspects and public systems of the participants to ensure that they were fully utilized and communicated with the available local resource managers to link them with the consent of the participants.

### 5.4. Local Resource Linkage

Researchers educated participants and caregivers on stroke-related information to enhance their understanding of stroke. This training was provided to individuals by referring to the health information bulletin board data distributed by the Central Health & Medical Center for Persons with Disabilities and the National Rehabilitation Center.

### 5.5. Task Fulfillment Rate

The researcher provided task notes to identify participants' difficulties in performing tasks. Referring to this, the task fulfillment rate was analyzed. As a result of calculating based on the intervention period, the task fulfillment rates each among the 1, 2, and 3 participants were 95%, 100%, and 97%.

## 6. Dependent Variable

### 6.1. Session-Dependent Variable (Frequency of Occupational Performance Skill Change)

In this study, based on the AMPS skills definition used by Fisher and Bray Jones [20], the occupational performance skills were operatively defined based on the three techniques of coordinates, sequences, and heeds. Two occupational therapists with more than five years of clinical trials recorded the frequency of occupational performance that decreased or effectively showed physical effort and conducted occupational performance analysis.

The article "The Effects of Occupation-Based Community Rehabilitation for Improving Activities of Daily Living and Health-Related Quality of Life of People with Disabilities after Stroke Living at Home: A Single Subject Design" was published in 2022. Journal: Occup Ther Int.

As shown in Table 1, the operational definitions of occupational performance skills are listed.

### 6.2. Pre- and Postintervention-Dependent Variables

#### 6.2.1. Changes in the Quality of Occupational Performance

We measured the quality of occupational performance evaluating the AMPS and analyzed using OTAPS (Occupational Therapy Assessment Package software). The AMPS task code was applied differently for each participant. The task codes of participant 1 before the start of the study were beverage from the refrigerator-one person (A1) and making a freestanding bed, “duvet” edges folded under (K3), after the end of the intervention period upper and lower body dressing-garments stored (P7), and instant noodles, soup, or beans-one person (I8). The task codes of participant 2 before the start of the study were upper body dressing-garment within reach (P6) and making a freestanding bed, “duvet” edges folded under (K3), after the end of the intervention period boiled/brewed coffee or tea and cookies/biscuits served at a table-two to four persons (G1), and heating a precooked meal or dessert in a microwave-one or two persons (I18). The task codes of participant 3 before the start of the study were heating a precooked meal or dessert in a microwave-one or two persons (I18) and pot of boiled/brewed coffee or tea-one or two persons (A3) and after the end of the intervention period rice, soup, and a side dish-one person (I22), and cleaning a bathroom (J7).

#### 6.2.2. Change in the Quality of Life

Participants' quality of life was measured through EQ-5D. The evaluation was conducted for 4 weeks before the start of the study, after the end of the intervention period, and after the end of the intervention.

## 7. Data Analysis

The frequency of efficient occupational performance that appears during daily task performance for each session was recorded numerically, and the standard deviation of baseline A and the average value was visually analyzed through a linear graph and two standard deviation (2SD) bands. AMPS, MBI, and EQ-5D results were evaluated in the pre, post, and subsequent stages. As for the dependent variable for each session, the frequency of occupational performance skills in daily life was analyzed using the results of the researcher.

The article "The Effects of Occupation-Based Community Rehabilitation for Improving Activities of Daily Living and Health-Related Quality of Life of People with Disabilities after Stroke Living at Home: A Single Subject Design" was published in 2022. Journal: Occup Ther Int.

## 8. Results

### 8.1. Participants

The general characteristics of participants are illustrated by Table 2, and three participants completed the study.

## 9. Changes in the Frequency of Occupational Performance Skills for Each Session

### 9.1. Changes in Coordinates Frequency

As can be seen in Figure 1, participant 1 showed an increase of 607% from an average of 1.4 (range: 0-2) to an average of 8.5 (range: 1-15) after the intervention phase was applied during the baseline phase A, an average of 13.2 (range: 12-14) during the baseline phase A', and 12 during the follow-up phase after 4 weeks. Participant 2 showed an increase of 388% from an average of 1.4 (range: 1-2) to an average of 5.4 (range: 3-8) after the intervention phase was applied during the baseline phase A, an average of 7 (range: 6-8) during the baseline phase A', and 7 during the follow-up phase after 4 weeks. Participant 3 was seen an increase of 327% from an average of 3.8 (range: 3-5) to an average of 12.4 (range: 7-18) after the intervention phase was applied during the baseline phase A, an average of 14.8 (range: 13-16) during the baseline phase A', and 15 during the follow-up phase after 4 weeks.

### 9.2. Changes in Sequences Frequency

As can be seen in Figure 2, participant 1 showed an increase of 275% from an average of 6.4 (range: 5-8) to an average of 17.6 (range: 8-25) after the intervention phase was applied during the baseline phase A, an average of 22 (range: 21-23) during the baseline phase A', and 21 during the follow-up phase after 4 weeks. Participant 2 showed an increase of 377% from an average of 3.6 (range: 3-5) to an average of 13.6 (range: 8-18) after the intervention phase was applied during the baseline phase A, an average of 14.2 (range: 13-15) during the baseline phase A', and 14 during the follow-up phase after 4 weeks. Participant 3 was seen an increase of 233% from an average of 8.4 (range: 8-9) to an average of 19.6 (range: 13-25) after the intervention phase was applied during the baseline phase A, an average of 24 (range: 23-25) during the baseline phase A', and 25 during the follow-up phase after 4 weeks.

### 9.3. Changes in Heeds Frequency

As can be seen in Figure 3, participant 1 showed an increase of 379% from an average of 2.6 (range: 2-3) to an average of 9.9 (range: 5-15) after the intervention phase was applied during the baseline phase A, an average of 12.4 (range: 11-13) during the baseline phase A', and 12 during the follow-up phase after 4 weeks. Participant 2 showed an increase of 47% from an average of 1.6 (range: 0-4) to an average of 8.4 (range: 4-11) after the intervention phase was applied during the baseline phase A, an average of 9.6 (range: 8-11) during the baseline phase A', and 11 during the follow-up phase after 4 weeks. Participant 3 was seen an increase of 188% from an average of 7 (range: 6-8) to an average of 13.1 (range: 8-16) after the intervention phase was applied during the baseline phase A, an average of 14 (range: 12-15) during the baseline phase A', and 14 during the follow-up phase after 4 weeks.

The article "The Effects of Occupation-Based Community Rehabilitation for Improving Activities of Daily Living and Health-Related Quality of Life of People with Disabilities after Stroke Living at Home: A Single Subject Design" was published in 2022. Journal: Occup Ther Int.

## 10. Changes in Pre-, Post-, and Follow-up Phases

### 10.1. Changes in Quality of Activities of Daily Living

The AMPS logit of participant 1 increased to motor skills 1.2 logit (0.4 to 1.6) and process skills 0.8 logit (0.8 to 1.6), and the most noticeable changes were stabilizes, bends, coordinates, paces, sequences, and heeds. The AMPS logit of participant 2 increased to motor skills 1.4 logit (0.2 to 1.8) and process skills 1.3 logit (0.4 to 1.7), and the most noticeable changes were aligns, reaches, coordinates, heeds, sequences, and terminates. The AMPS logit of participant 3 increased to motor skills 1.1 logit (0.7 to 1.8) and process skills 0.9 logit (0.9 to 1.8), and the most noticeable changes were grips, coordinates, endures, paces, heeds, and sequences.

### 10.2. Changes in Independent of Activities of Daily Living

The MBI score of participant 1 was changed from prephase 49 points (severe dependent) to postphase 72 points (moderate dependent). Like the postphase score, the follow-up phase score was 72 points, showing that the independence of daily life activities was well maintained. In activities, noticeable changes were seen in toilet, dressing, and chairs/bed transfer. The MBI score of participant 2 was changed from prephase 48 points (severe dependent) to postphase 76 points (mild dependent). Like the postphase score, the follow-up phase score was 76 points, showing that the independence of daily life activities was well maintained. In activities, conspicuous changes were presented in bathing, toilet, and chairs/bed transfer. The MBI score of participant 3 was changed from prephase 79 points (mild dependent) to postphase 95 points (minimal dependent). Like the postphase score, the follow-up phase score was 95 points, showing that the independence of daily life activities was well maintained. In activities, remarkable changes occurred in stair climbing, ambulation, and dressing.

### 10.3. Changes in Health-Related Quality of Life

Participant 1's EQ-5D score improved 0.043 points from 0.677 points in prephase to 0.72 points in postphase. The follow-up phase score also showed that the quality of life was well maintained with 0.72 points. Participant 2's EQ-5D score improved 0.254 points from 0.423 points in prephase to 0.677 points in postphase. The follow-up phase score also showed that the quality of life was well maintained with 0.677 points. Participant 3's EQ-5D score improved 0.25 points from 0.47 points in prephase to 0.72 points in postphase. The follow-up phase score also showed that the quality of life was well maintained with 0.72 points.

The article "The Effects of Occupation-Based Community Rehabilitation for Improving Activities of Daily Living and Health-Related Quality of Life of People with Disabilities after Stroke Living at Home: A Single Subject Design" was published in 2022. Journal: Occup Ther Int.

## 11. Discussion

The study was aimed at investigating the effects of occupation-based community rehabilitation on activities of daily living and health-related quality of life of people with disabilities after stroke at home. The purpose was to observe and analyze the activities of daily living of the participants for each session to observe changes in their occupational performance, to evaluate their activities of daily living and quality of life before and after intervention, and to understand their applicability to community-based rehabilitation.

As a result of applying occupation-based community rehabilitation, it was confirmed that all participants' activities of daily living and quality of life improved. In the case of MBI conducted during the pre-, post-, and follow-up periods, to minimize errors caused by interviews in the form of questionnaires, the performance of the remaining eight items excluding urine and fecal activity was directly observed and the trend of change was investigated. Plans could be made based on the participation's occupation, and activities of daily living scores were improved in all participants. In particular, in the case of participant 2, the use of the toilet has improved significantly from 2 points to 10 points. The reason for the improvement was that although he received total help from his caregiver due to fall anxiety, he was able to reduce anxiety, perform tasks with appropriate level, and acquire occupational skills.

This result is consistent with previous studies that show that participation's occupation-based methods improved their activities daily of living more than repeatedly learning normal patterns of stroke patients [23].

AMPS scores were expressed in logits, and changes powerful than 0.3 logits were clinically significant. As explained by the AMPS evaluation results, participants 1, 2, and 3 improved logit motor scores of 1.2, 1.6, and 1.1 and process scores of 0.8 points, 1.3 points, and 0.9 points, respectively. Coordinates, sequences, and heeds were improved in all participants. There are many studies showing that occupation-based community rehabilitation improves occupational performance [2, 6, 9, 24, 25].

The increase in activities of daily living of stroke patients and health-related quality of life are highly related, so it is necessary to examine them together. EQ-5D allows screening of participation's quality of life by Kang et al. [17]. All participants were found to have improved the EQ-5D. Participant 3 changed all items related to mobility, self-management, daily activities, and pain/inconvenience, and the postevaluation result was evaluated as 0.72 points, improving through occupation-based community rehabilitation. In this study, it was found that occupation-based community rehabilitation is important in improving the activities of daily living and health-related quality of life of stroke participants.

The article "The Effects of Occupation-Based Community Rehabilitation for Improving Activities of Daily Living and Health-Related Quality of Life of People with Disabilities after Stroke Living at Home: A Single Subject Design" was published in 2022. Journal: Occup Ther Int.

## 12. Limitations and Future Research

Since this study has a small number of cases, the correlation between each evaluation should also be studied. In addition, rehabilitation service variables other than occupation-based community rehabilitation were not controlled. There is a possibility that there has been a change in the overall lifestyle of the participant, the resulting good habits, and the influence of daily life. In future research, various data analyses using wearable devices, or the Internet of Things (IoT) should be combined to redesign the subject's lifestyle.

## 13. Conclusion

Through this study, it was possible to increase the independence of daily life and improve the quality of life related to health by applying occupational-based community rehabilitation to people with disabilities living at home after stroke. The occupational-based community rehabilitation consisted of a series of processes, including an occupational therapy intervention process model.

The results of this study are as follows.

First, after applying occupational-based community rehabilitation, the activities of daily living of all participants was improved, and the degree of independence of daily life improved.

Second, the applications for occupational community rehabilitation have been proven to have an crucial effect on the health-related quality of life of all participants.

Third, after the occupational community rehabilitation was applied, the quality of occupational performance improved. All three items performed by all participants made realistic changes possible. After the intervention phase was over, occupations were even well maintained.

## Figures and Tables

**Figure 1:** Changes in coordinates frequency.

**Figure 2:** Changes in sequences frequency.

**Figure 3:** Changes in heeds frequency.

**Table 1:** Operational definitions of occupational performance skills.

Occupational performance skills	Operational definition
Coordinates	Fix and manipulate objects with two parts of the task
Sequences	Perform the task according to the order discussed
Heeds	Complete the task as discussed

**Table 2:** General characteristics of the participants.

	Participant 1	Participant 2	Participant 3
Gender	Male	Female	Male
Age	58 y	37 y	59 y
Cause of disease	Cerebral hemorrhaged	Cerebral hemorrhaged	Cerebral infarction
Period of disease	2017/11	2017/7	2019/4
Duration of disease	29 m	33 m	12 m
Types of disabilities	Brain lesion	Brain lesion	Brain lesion
Amount of disabilities	Severe	Severe	Severe
Impaired side	Left	Left	Right
Sensory	Normal	Normal	Normal
Chronic diseases	High blood pressure, diabetes	Low blood pressure	High blood pressure, diabetes
Caregiver	Wife	Mother	Assistant worker
Dominant hand	Right	Right	Right
Assistive device	AFO	W/C	Quad cane
Job	Luxury goods salesman	English teacher	Taxi driver
Desire to occupation	Shopping	Travel	Getting a job
MBI	49	46	79
EQ-5D	0.677	0.423	0.47
AMPS			
Motor skills	0.4	0.2	0.7
Process skills	0.8	0.4	0.9
MMSE-K	24	21	24

AMPS: Assessment of Motor and Process Skills, EQ-5D: EuroQol-5 Dimension, MBI: Modified Barthel Index, MMSE-K: Mini-Mental State Examination.

The article "The Effects of Occupation-Based Community Rehabilitation for Improving Activities of Daily Living and Health-Related Quality of Life of People with Disabilities after Stroke Living at Home: A Single Subject Design" was published in 2022. Journal: Occup Ther Int.

## Data Availability

The data used to support the findings of this study are available from the corresponding author upon request.

## References

[1] Almhdawi K., Mathiowetz V., White M., Delmas R. (2016). Efficacy of occupational therapy task-oriented approach in upper extremity post-stroke rehabilitation. *Occupational Therapy International*.

[2] Yoon J. A. (2011). *Effects of Basic IQ and Executive IQ on ADL in Stroke Patients, [Ph.D. thesis]*.

[3] Kim J. H., Kang H. S., Kim W. O., Wang M. J., Chang C. M. (2006). Factors affecting the quality of life in stroke patient at home. *The Korean Journal of Rehabilitation Nursing*.

[4] Eskandar M. E., Otadi M., Mojibi T. (2018). Ranking the desirability indicators of community-based rehabilitation (CBR) based on analytical hierarchy process. *International Journal of Psychology and Behavioral Sciences*.

[5] Hammel J., Jones R., Gossett A., Morgan E. (2006). Examining barriers and supports to community living and participation after a stroke from a participatory action research approach. *Topics in Stroke Rehabilitation*.

[6] Moon K. T., Park H. Y., Kim J. B. (2020). The effects of occupation-based community rehabilitation for improving occupational performance skills and activity daily living of stroke home disabled people: a single subject design. *Therapeutic Science for Rehabilitation*.

[7] Ministry of Health and Welfare 2019 study on the disabled. https://www.data.go.kr/dataset/15004328/fileData.do.

[8] An T. G., Kim K. U. (2016). Need on homebased occupational therapy and caregiving burden: Busan and south Gyeongsang areas centered around. *Journal of Humanities and Social Science*.

[9] Choi H. S. (2002). Effects of a community based rehabilitation program on cognitive status, ADLP, and occupational performance/satisfaction of old CVA patients. *論文集-東南保健大學*.

The article "The Effects of Occupation-Based Community Rehabilitation for Improving Activities of Daily Living and Health-Related Quality of Life of People with Disabilities after Stroke Living at Home: A Single Subject Design" was published in 2022. Journal: Occup Ther Int.

[10] Jang W. H. (2020). *A Study on Job Analysis and Guidelines Development of Community Based Home Visit Ocupational Therapists*.

[11] Lee H. Y., Sagong B. (2015). The effect of home based rehabilitation program on activities of daily living, self-efficacy, quality of life among chronic stroke patients. *Journal of Special Education & Rehabilitation*.

[12] Arya K. N., Verma R., Garg R. K., Sharma V. P., Agarwal M., Aggarwal G. G. (2012). Meaningful task-specific training (MTST) for stroke rehabilitation: a randomized controlled trial. *Topics in Stroke Rehabilitation*.

[13] Keglovits M., Somerville E., Stark S. (2015). In-home occupational performance evaluation for providing assistance (I-HOPE assist): an assessment for informal caregivers. *American Journal of Occupational Therapy*.

[14] De Coninck L., Bekkering G. E., Bouckaert L., Declercq A., Graff M. J., Aertgeerts B. (2017). Home- and community-based occupational therapy improves functioning in frail older people: a systematic review. *Journal of the American Geriatrics Society*.

[15] Newell J. M., Lyons R., Martin-Misener R., Shearer C. L. (2009). Creating a supportive environment for living with stroke in rural area: two low-cost community-based interventions. *Topics in Stroke Rehabilitation*.

[16] Hsueh I. P., Lin J. H., Jeng J. S., Hsieh C. L. (2002). Comparison of the psychometric characteristics of the functional independence measure, 5 item Barthel index, and 10 item Barthel index in patients with stroke. *Journal of Neurology, Neurosurgery & Psychiatry*.

[17] Kang E. J., Shin H. S., Park H. J., Jo M. W., Kim N. Y. (2006). A valuation of health status using EQ-5D. *Korean Journal of Health Economics and Policy*.

[18] Lee Y. K., Nam H. S., Chuang L. H. (2009). South Korean time trade-off values for EQ-5D health states: modeling with observed values for 101 health states. *Value in Health*.

[19] Fisher A. G. (2014). Occupation-centred, occupation-based, occupation-focused: same, same or different?. *Scandinavial Journal of Occupational Therapy*.

[20] Fisher A. G., Bray Jones K. (2014). *Assessment of Motor and Process Skills, vol. 2*.

[21] Thivierge S., Simard M., Jean L., Grandmaison É. (2008). Errorless learning and spaced retrieval techniques to relearn instrumental activities of daily living in mild Alzheimer’s disease: a case report study. *Neuropsychiatric Disease and Treatment*.

[22] Jo H., Choi Y. J., Shin M. K. (2013). The influence of home modification on ADL performance of the elderly in residential environment. *Journal of Korean Society of Assistive Technology*.

The article "The Effects of Occupation-Based Community Rehabilitation for Improving Activities of Daily Living and Health-Related Quality of Life of People with Disabilities after Stroke Living at Home: A Single Subject Design" was published in 2022. Journal: Occup Ther Int.

[23] Yang Y. R., Wang R. Y., Lin K. H., Chu M. Y., Chan R. C. (2006). Task-oriented progressive resistance strength training improves muscle strength and functional performance in individuals with stroke. *Clinical Rehabilitation*.

[24] Skubik-Peplaski C., Custer M., Powell E., Westgate P. M., Sawaki L. (2017). Comparing occupation-based and repetitive task practice interventions for optimal stroke recovery: a pilot randomized trial. *Physical & Occupational Therapy In Geriatrics*.

[25] Shah S., Vanclay F., Cooper B. (1989). Improving the sensitivity of the Barthel index for stroke rehabilitation. *Journal of Clinical Epidemiology*.

